RETRACTED

# Long non-coding RNA XIST promotes cell growth and metastasis through regulating miR-139-5p mediated Wnt/β-catenin signaling pathway in bladder cancer

**DOI:** 10.18632/oncotarget.21791

**Published:** 2017-10-10

**Authors:** Yangyang Hu, Chao Deng, He Zhang, Jing Zhang, Bo Peng, Chuanyi Hu

**Affiliations:** ^1^ Department of Urology, Gongli Hospital, The Second Military Medical University, Shanghai 200135, China; ^2^ Department of First Clinical Medical College, Nanjing Medical University, Nanjing 211166, China

**Keywords:** lncRNA, XIST, bladder cancer, miR-139-5p, Wnt1

## Abstract

Bladder cancer is one of the most common urological malignancy all over the world. Recently, long non-coding RNA (lncRNA) XIST has been identified as an oncogenic gene in several type of cancers. However, the expression level and functional role of XIST in bladder cancer remain largely unknown. In the present study, we found that XIST was significantly up-regulated in bladder cancer tissues and cell lines, and was correlated with poor prognosis of bladder cancer patients. Furthermore, XIST knockdown significantly inhibited bladder cancer cell growth and metastasis *in vitro* and tumor growth *in vivo*. We also demonstrated that XIST acted as a competing endogenous RNA for miR-139-5p and repression of miR-139-5p could restore the inhibitory effects on bladder cancer cells induced by XIST shRNA. In addition, we identified that Wnt1 was a direct target of miR-139-5p, and XIST played the oncogenic role in bladder cancer by activating the Wnt/β-catenin signaling pathway. Taken together, our study suggested that lncRNA XIST may serve as a prognostic biomarker and a potential therapeutic target for bladder cancer.

## INTRODUCTION

Bladder cancer is one of the most common urological malignancy all over the world [1]. For the moment, surgical resection and chemotherapy remain the curative strategies for bladder cancer treatment [2]. Despite there have been great improvements in current clinical treatment for bladder cancer such as adjuvant chemo-radiotherapies and immunological therapy, the five-year overall survival rate is far from satisfactory [3–5]. Therefore, it is urgent need to explore the molecular mechanisms underlying bladder cancer tumorigenesis and progression to discover novel molecular biomarkers and therapeutic strategies for bladder cancer.

Long non-coding RNAs (lncRNAs), a class of non-coding RNAs with more than 200 nucleotides in length [6], have been reported to involve in a large range of biological processes, including transcriptional regulation, cell differentiation, proliferation, and tumorigenesis [7, 8]. Recent emerging evidences have shown that lncRNAs play important roles in the development of human diseases, especially in cancers [9, 10].

RETRACTED

X-inactive specific transcript (XIST) is a kind of lncRNA derived from XIST gene and the crucial regulator of X inactivation in mammals [11]. According to recent studies, XIST is up-regulated in several cancers, including hepatocellular carcinoma [12], gastric cancer [13], non-small cell lung cancer [14], glioma [15], and pancreatic cancer [16], the overexpression of XIST is highly associated with growth, invasion, and metastasis of these cancers. For instance, XIST was up-regulated in gastric cancer tissues and cell lines, and knockdown of XIST exerted tumor-suppressive effects by inhibiting cell proliferation, migration and invasion [17]. However, the expression and underlying molecular mechanism of XIST in bladder cancer remain largely unknown.

MicroRNAs (miRNAs), a group of short noncoding RNA molecules with 18-25 nucleotides in length, participate in multiple cellular processes at the posttranscriptional level by binding to the 3’-untranslated region (UTR) of messenger RNA (mRNA), resulting in mRNA degradation or translation repression [18]. Accumulating evidences have demonstrated that the dysfunction of miRNA play a critical role in cancer initiation and development [19, 20]. LncRNAs exert their functions through different mechanisms, a new described regulatory mechanism that lncRNAs may act as molecular sponges of miRNAs [21]. For example, Song et al reported that XIST functioned as an oncogene in human nasopharyngeal carcinoma through sponging miR-34a-5p [22]. However, the interaction between XIST and miRNA in bladder cancer has not been studied up to now.

In this study, we first detected the expression of XIST in bladder cancer by using real-time PCR and found that XIST was significantly up-regulated and closely correlated with the advanced progression of bladder cancer. Furthermore, we explored the biological roles of XIST in bladder cancer both *in vitro* and *in vivo*, and demonstrated that XIST functions as a sponge of miR-139-5p to regulate the expression of Wnt1 and activity of the Wnt/β-catenin signaling pathway, thus acting as an oncogene in pathogenesis of bladder cancer. These results provide the evidence that the regulatory mechanism of newly identified lncRNA XIST/miR-139-5p/Wnt1 axis in carcinogenesis and metastasis of bladder cancer, which may shed new light on lncRNA-directed applications in cancer diagnosis and therapy.

## RESULTS

### XIST expression is up-regulated in bladder cancer tissues and cell lines, and correlates with poor prognosis

The relative expression levels of XIST in 52 pairs of bladder cancer tissues and adjacent non-tumor tissues was firstly detected by qRT-PCR. The fold change of XIST expression levels (bladder cancer tissues/adjacent non-tumor tissues) in each patient was indicated in Figure 1A. As shown in Figure 1B, XIST expression was significantly up-regulated in bladder cancer tissues compared with adjacent non-tumor tissues. Moreover, the relative expression of XIST was significantly higher in patients with advanced tumor stage, large tumor size, high histological grade and lymph nodal metastasis (Figure 1C-1F). We then analyzed the correlations between XIST expression and clinicopathological characteristics of bladder cancer patients. The results indicated that high expression levels of XIST was correlated with advanced tumor stage, large tumor size, high histological grade and lymph nodal metastasis, while was not correlated with age, gender and multiplicity (Table 1). The expression levels of XIST in bladder cancer cell lines (T24, 5637, EJ, UMUC3 and J82) were also significantly up-regulated compared to normal urothelial cells SV-HUC-1 (Figure 1G).

RETRACTED

**Figure 1:** XIST was up-regulated in bladder cancer tissues and cell lines, and related to overall survival **(A)** The heights of the columns in the chart represented the log2-transformed fold changes (bladder cancer tissues/normal tissues) in XIST expression in 52 patients with bladder cancer. **(B)** The relative expression levels of XIST was significantly up-regulated in bladder cancer tissues compared to adjacent normal tissues. **(C-F)** The relative expression levels of XIST was higher in patients with advanced tumor stage, high histological grade, lymph nodal metastasis and tumor size, respectively. **(G)** The relative expression levels of XIST was significantly up-regulated in bladder cancer cell lines compared to normal urothelial cells. **(H)** Correlation between XIST expression and overall survival of patients with bladder cancer by Kaplan-Meier analysis. Data are shown as mean ± SD. *P < 0.05, **P < 0.01, ***P < 0.001.

**Table 1:** Correlation between lncRNA XIST expression and clinicopathological characteristics of bladder cancer patients

Parameters	XIST expression		P value
	High (n=32)	Low (n=20)	
Age (years)			0.540
> 60	18	12	
≤ 60	14	8	
Gender			0.658
Male	20	13	
Female	12	7	
TNM stage			0.012*
T1/T2	19	15	
T3/T4	13	5	
Tumor size (cm)			0.028*
> 3	24	11	
≤ 3	8	9	
Histological grade			0.036*
High	22	10	
Low	10	10	
Lymph node metastasis			0.042*
Negative	18	18	
Positive	14	2	
Multiplicity			0.425
Single	17	12	
Multiple	15	8	

*P<0.05 was considered significant (Chi-square test between two groups).

In addition, the prognostic value of XIST expression was determined for overall survival in bladder cancer patients by the Kaplan-Meier analysis. Result revealed that high expression level of XIST was significantly correlated with shorter overall survival (Figure 1H).

RETRACTED

### Knockdown of XIST inhibits cell proliferation, induces cell cycle arrest and apoptosis in bladder cancer cells

To further investigate the possible biological roles of XIST in bladder cancer *in vitro*, we knockdown the expression of XIST in bladder cancer cells (T24 and 5637) by shRNA. The efficiency of XIST knockdown was subsequently confirmed by qRT-PCR, and the sh-XIST-2 had a better knockdown efficiency for XIST, which was used in the following experiments (Figure 2A). We firstly evaluated the effects of XIST knockdown on bladder cancer cell growth. CCK-8 assay indicated that XIST knockdown significantly inhibited cell proliferation of both T24 and 5637 cells compared with negative control (Figure 2B and 2C). In addition, results from colony formation assay revealed that the number of colonies in cells transfected with sh-XIST were obviously lower than in cells transfected with sh-NC (Figure 2D).

**Figure 2:** Knockdown of XIST inhibited cell proliferation, induced cell cycle arrest and promoted cell apoptosis in bladder cancer cells **(A)** XIST expression was significantly down-regulated by transfection of XIST shRNA in T24 and 5637 cells. **(B** and **C)** CCK-8 assays showed that XIST knockdown inhibited cell proliferation in bladder cancer cells. **(D)** Colony formation assays indicated that XIST knockdown reduced the number of colonies. **(E)** XIST knockdown induced cell cycle arrest at G0/G1 phase in T24 and 5637 cells by flow cytometry. **(F)** XIST knockdown led to a remarkable increase of the percentage of apoptotic cells. Data are shown as mean ± SD. *P < 0.05, **P < 0.01.

Next, flow cytometric analysis was performed to determine the cell cycle distribution and apoptosis in bladder cancer cells. Cell cycle assay showed that XIST knockdown induced cell cycle arrest at G0/G1 phase in both T24 and 5637 cells compared with negative control (Figure 2E). Cell apoptosis analysis demonstrated that transfection of sh-XIST led to a remarkable increase of the percentage of apoptotic cells (Figure 2F). Taken together, these results suggested that knockdown of XIST expression inhibited bladder cancer cell proliferation by inducing cell cycle arrest and promoting cell apoptosis.

### Knockdown of XIST inhibits cell migration and invasion in bladder cancer cells

To investigate the influence of XIST knockdown on migration and invasion of bladder cancer cells, we performed transwell assays in T24 and 5637 cells. By cell migration assay, we found XIST knockdown obviously inhibited the migratory ability of bladder cancer cells compared with negative control (Figure 3A). In addition, cell invasion assay showed that the invasive ability of bladder cancer cells was significantly suppressed by XIST knockdown (Figure 3B). Collectively, these findings clearly indicated that knockdown of XIST expression suppressed cell metastasis in bladder cancer cells.

RETRACTED

**Figure 3:** Knockdown of XIST inhibited cell migration and invasion in bladder cancer cells **(A)** The migratory ability of bladder cancer cells transfected with XIST shRNA was significantly inhibited by trans-well assay. **(B)** The invasive ability of bladder cancer cells transfected with XIST shRNA was significantly inhibited by trans-well assay. Data are shown as mean ± SD. *P < 0.05.

### XIST directly interacts with miR-139-5p

Recently, increasing studies have demonstrated that lncRNAs can act as competitive endogenous RNAs (ceRNAs) of miRNAs, and in turn regulating their biological functions. Through online bioinformatics database (starBase v2.0), we predicted miR-139-5p contained putative binding sites with XIST (Figure 4A). To confirm whether XIST was a functional target of miR-139-5p, a dual-luciferase reporter assay was performed. Our results demonstrated that miR-139-5p significantly decreased the luciferase activity of luciferase reporter vector XIST-WT in HEK293T cells, while did not change the luciferase activity of XIST-MUT (Figure 4B). In addition, XIST knockdown strongly increased the relative expression levels of miR-139-5p in T24 and 5637 cells (Figure 4C). However, there was no obvious change in the XIST expression after transfection with miR-139-5p mimics in bladder cancer cells (Figure 4D). To further investigate whether XIST and miR-139-5p binding together, RNA pull-down assay was conducted in HEK293T cells. We found XIST could pull-down miR-139-5p, the antisense strand of XIST probe was used as negative control (Figure 4E).

**Figure 4:** XIST directly interacted with miR-139-5p in bladder cancer cells **(A)** Bioinformatics analysis showed the predicted binding sites between XIST and miR-139-5p. **(B)** Luciferase reporter assay demonstrated that miR-139-5p overexpression significantly decreased the luciferase activity of XIST-WT in HEK293T cells. **(C)** XIST knockdown increased the relative expression of miR-139-5p in T24 and 5637 cells. **(D)** There was no obvious change in XIST expression after transfection with miR-139-5p mimics in T24 and 5637 cells. **(E)** XIST could pull-down miR-139-5p expression in HEK293T cells by RNA pull-down assay. **(F)** The relative expression levels of miR-139-5p was significantly down-regulated in bladder cancer tissues compared to adjacent normal tissues. **(G)** The relative expression levels of miR-139-5p was significantly down-regulated in bladder cancer cell lines compared to normal urothelial cells. **(H)** Correlation analysis indicated the negative relationship between XIST and miR-139-5p expression in bladder cancer tissues. Data are shown as mean ± SD. *P < 0.05, **P < 0.01, ***P < 0.001.

RETRACTED

Next, the relative expression levels of miR-139-5p in bladder cancer tissues and cell lines were detected. MiR-139-5p expression were significantly down-regulated in bladder cancer tissues and cell lines compared with adjacent non-tumor tissues and normal urothelial cells (Figure 4F and 4G). Furthermore, an inverse correlation was found between XIST expression and miR-139-5p expression in bladder cancer tissues by Pearson’s correlation analysis (Figure 4H). These results demonstrated that XIST could directly interact with miR-139-5p in bladder cancer.

### XIST regulates bladder cancer cell growth and metastasis through miR-139-5p

Our previous results indicated that XIST knockdown could act as tumor suppressive roles in bladder cancer progression, and XIST was a direct target of miR-139-5p. We further investigate whether XIST exerts biological functions in bladder cancer cells through miR-139-5p. MiR-139-5p inhibitor was transfected into T24 and 5637 cells stably co-transfected with XIST shRNA or negative control. CCK-8 and colony formation assays revealed that the inhibition of cell proliferation induced by XIST knockdown was significantly reversed by miR-139-5p inhibitor (Figure 5A-5C). Flow cytometric analysis demonstrated that XIST knockdown obviously induced cell cycle arrest at G0/G1 phase and promoted cell apoptosis in T24 and 5637 cells, which were largely abolished by miR-139-5p inhibitor (Figure 5D and 5E). In addition, repression of miR-139-5p in T24 and 5637 cells could restore the reduced abilities of cell migration and invasion caused by XIST shRNA (Figure 5F and 5G). Taken together, these data suggested that XIST knockdown suppressed bladder cancer cell growth and metastasis through miR-139-5p.

**Figure 5:** Repression of miR-139-5p restored the inhibitory effects on bladder cancer cells induced by XIST knockdown **(A-C)** The inhibitory effect of XIST knockdown on cell proliferation in T24 and 5637 cells could be restored by miR-139-5p inhibition by CCK-8 assay and colony formation assay. **(D)** Flow cytometric analysis showed that XIST knockdown induced cell cycle arrest at G0/G1 phase in T24 and 5637 cells, which was largely abolished by miR-139-5p inhibitor. **(E)** XIST knockdown promoted cell apoptosis, while co-transfected with miR-139-5p inhibitor could reverse this change. **(F** and **G)** The inhibitory effect of XIST knockdown on cell migration and invasion could be reversed by miR-139-5p inhibition by trans-well assays. Data are shown as mean ± SD. *P < 0.05, **P < 0.01.

RETRACTED

### MiR-139-5p inactivates the Wnt/β-catenin signaling pathway via directly targeting Wnt1

Through online bioinformatics database (TargetScan), we found Wnt1 was a potential downstream target of miR-139-5p (Figure 6A). To further confirm the direct interaction between Wnt1 and miR-139-5p, a dual-luciferase reporter assay was performed in HEK293T cells. Our results showed that miR-139-5p mimics led to a significant decrease of the luciferase activity of Wnt1-WT, but could not change the luciferase activity of Wnt1-MUT (Figure 6B). The expression levels of Wnt1 in T24 and 5637 cells transfected with miR-139-5p mimics were examined by qRT-PCR and western blot analysis. MiR-139-5p overexpression remarkably inhibited the mRNA and protein expression levels of Wnt1 (Figure 6C and 6D).

**Figure 6:** MiR-139-5p inactivated the Wnt/β-catenin signaling pathway through directly targeting Wnt1 **(A)** Bioinformatics analysis showed the predicted binding sites between miR-139-5p and Wnt1. **(B)** Luciferase reporter assay demonstrated that miR-139-5p overexpression significantly decreased the luciferase activity of Wnt1-WT in HEK293T cells. **(C)** MiR-139-5p overexpression decreased the mRNA expression of Wnt1 in T24 and 5637 cells by qRT-PCR assay. **(D)** The protein expression levels of tumor-related genes (Wnt1, β-catenin, and cyclin-D1) in the Wnt/β-catenin signaling pathway were suppressed in T24 and 5637 cells by miR-139-5p overexpression by western blot assay. Data are shown as mean ± SD. *P < 0.05, **P < 0.01.

Subsequently, we explored whether miR-139-5p could affect the Wnt/β-catenin signaling pathway, which was broadly involved in the process of promoting tumorigenesis and EMT induction [23, 24]. Western blot analysis was conducted to detect the protein expression levels of β-catenin and cyclin-D1. Our data indicated that β-catenin and cyclin-D1 expressions were also significantly inhibited by the up-regulation of miR-139-5p in T24 and 5637 cells. These data demonstrated that miR-139-5p was able to inactivate the Wnt/β-catenin signaling pathway through directly targeting Wnt1.

### XIST regulates the Wnt/β-catenin signaling pathway through miR-139-5p

We further investigated whether the Wnt/β-catenin signaling pathway was regulated by XIST, and whether this regulation was dependent on miR-139-5p. XIST shRNA or negative control were transfected into T24 and 5637 cells, whereafter co-transfected with miR-139-5p inhibitor. As expected, knockdown of XIST decreased the protein levels of Wnt1, β-catenin and cyclin-D1 in bladder cancer cells, while down-regulation of miR-139-5p could restore this repression (Figure 7A). QRT-PCR assay indicated that the mRNA expression of Wnt1 in 52 bladder cancer tissues was significantly up-regulated compared to adjacent non-tumor tissues (Figure 7B). We then tested the correlation between the expression levels of XIST, miR-139-5p, and Wnt1 in clinical tumor samples. It was found that XIST expression was positively correlated with Wnt1 expression, while miR-139-5p expression was negatively correlated with Wnt1 expression, respectively (Figure 7C and 7D). Taken together, these results suggested that XIST positively regulated the Wnt/β-catenin signaling pathway through miR-139-5p.

RETRACTED

**Figure 7:** XIST positively regulated the Wnt/β-catenin signaling pathway through miR-139-5p **(A)** The inhibitory effect of XIST knockdown on the protein expression levels of Wnt1, β-catenin, and cyclin-D1 in T24 and 5637 cells could be restored by miR-139-5p inhibition. **(B)** The relative expression levels of Wnt1 mRNA was significantly up-regulated in bladder cancer tissues compared to adjacent normal tissues. **(C** and **D)** XIST expression was positively correlated with Wnt1 expression in bladder cancer tissues, while miR-139-5p expression was negatively correlated with Wnt1 expression. *P < 0.05.

### XIST inhibition suppresses bladder cancer cell proliferation *in vivo*

To further evaluate the functional role of XIST in tumor growth of bladder cancer *in vivo*, XIST shRNA or negative control stably transfected T24 cells were injected into nude mice. Knockdown of XIST significantly decreased the tumor volumes and weights compared with negative control group (Figure 8A-8C). Moreover, the relative expression of XIST and Wnt1 were significantly downregulated in tumor tissues of nude mice with XIST shRNA compared to negative control, and the relative expression of miR-139-5p was upregulated (Figure 8D). Ki-67 staining was performed to measure the cell proliferation in tumor tissues of nude mice, the results showed that knockdown of XIST inhibited tumor cell proliferation (Figure 8E). Accordingly, these data demonstrated that XIST knockdown suppressed tumor growth of bladder cancer *in vivo*.

**Figure 8:** XIST inhibition suppressed tumor growth of bladder cancer *in vivo* **(A)** Tumors collected from nude mice were excised. **(B** and **C)** The mean tumor volume and tumor weight of nude mice were suppressed in XIST shRNA group. **(D)** The relative expression levels of XIST, miR-139-5p and Wnt1 in tumor tissues of nude mice was examined by qRT-PCR. **(E)** Knockdown of XIST significantly decreased the percentage of Ki-67 positive cells in tumors of nude mice. Data are shown as mean ± SD. *P < 0.05, **P < 0.01, ***P < 0.001.

RETRACTED

## DISCUSSION

Accumulating evidence have reported that XIST could play critical roles in tumor progression of many human malignant cancers [25]. For example, Yao et al indicated that XIST expression was up-regulated in glioma tissues and human glioblastoma stem cells, moreover, knockdown of XIST exerted tumor-suppressive functions by inhibiting cell proliferation, migration and invasion as well as promoting apoptosis [26]. Wu et al demonstrated that high XIST expression predicted poor prognosis of patients with esophageal squamous cancer (ESCC), and XIST promoted malignant progression of ESCC through regulation of miR-101/EZH2 axis [27]. However, the clinical significance as well as underlying mechanism of XIST in bladder cancer are still unclear.

In this study, we found XIST expression was significantly up-regulated in bladder cancer tissues and cell lines compared with adjacent non-tumor tissues and normal urothelial cells. High expression level of XIST in patients with bladder cancer was correlated with advanced tumor stage, large tumor size, high histological grade, lymph nodal metastasis, and shorter overall survival. Furthermore, the biological function of XIST in bladder cancer was investigated. Our results indicated that knockdown of XIST expression markedly inhibited cell proliferation, migration, and invasion, induced cell cycle arrest and promoted apoptosis in bladder cancer cell lines. In addition, XIST inhibition suppressed tumor growth of bladder cancer *in vivo*. These data suggested that XIST acted as an oncogene in bladder cancer progression.

Recently, lncRNAs have been shown to function as natural miRNA sponges, in turn modulating the expression of miRNA. For example, Xu et al demonstrated that long non-coding RNA TUSC7 was a potential tumor suppressor in colorectal cancer (CRC), and TUSC7 could inhibit CRC cell proliferation by sponging miR-211-3p [28]. Huang et al showed that long non-coding RNA PVT1 functioned as a competing endogenous RNA by sponging miR-186 in gastric cancer, and promoted gastric cancer cell proliferation and invasion [29]. However, little is known about the relationship between lncRNA and miRNA in the carcinogenesis of bladder cancer. In the present study, we identified miR-139-5p as an inhibitory target of XIST by bioinformatics analysis and luciferase reporter assay. XIST knockdown could enhance the expression levels of miR-139-5p in bladder cancer cell lines, and further Pearson correlation analysis revealed a remarkably negative correlation between XIST expression and miR-139-5p expression in bladder cancer tissues. These results demonstrated that XIST acted as a molecular sponge of miR-139-5p in bladder cancer.

RETRACTED

MiRNAs may function as oncogenes or tumor suppressors in a variety of cellular processes during tumor formation [30]. A number of studies have suggested that miR-139-5p is a potential regulatory miRNA, which is usually down-regulated in malignant tumors including colorectal cancer, non-small cell lung cancer, ovarian cancer and bladder cancer [31–34]. Our study found that miR-139-5p expression was significantly decreased in bladder cancer tissues and cell lines, which was consistent with the results of previous research. Furthermore, repression of miR-139-5p could restore the inhibitory effects on bladder cancer cell proliferation and invasion by XIST knockdown. Having indicated the critical role of miR-139-5p in bladder cancer progression, we then searched for the potential gene effector involved in its function. Wnt1, a member from WNT gene family, functioned as an oncogene in several types of cancer [35, 36]. Recent study found that Wnt1 expression was significantly higher in cutaneous squamous cell carcinoma samples than in normal skin cells, moreover, Wnt1 expression was correlated with the histopathological differentiation [37]. Chen et al showed that overexpression of miRNA-148a inhibited migration and invasion of lung cancer cells, while knockdown of Wnt-1 had the similar effects of miRNA-148a overexpression, they suggested that miRNA-148a inhibited cell migration and invasion through targeting Wnt1 in non-small cell lung cancer [38]. We confirmed that miR-139-5p regulated the expression of Wnt1 in bladder cancer cells through directly targeting the 3’UTR of Wnt1. And an inverse correlation between miR-139-5p expression and Wnt1 expression in bladder cancer tissues was observed.

The Wnt/β-catenin signaling pathway played a crucial role in regulating a variety of biological processes, including cell proliferation, apoptosis, invasion, and differentiation [39]. It has been reported that aberrant activation of the Wnt/β-catenin signaling pathway was related to the initiation and progression of human cancers [40]. For example, Niu et al demonstrated that PPA1 silencing inhibited human epithelial ovarian cancer migration, EMT and metastasis by suppressing the Wnt/β-catenin signaling pathway [41]. Yang et al showed that FOXP3 promoted tumor growth and metastasis through activating the Wnt/β-catenin signaling pathway in non-small cell lung cancer [23]. In the present study, overexpression of miR-139-5p also led to significant decrease in the protein expression levels of β-catenin and cyclin-D1 in T24 and 5637 cells. Therefore, we concluded that miR-139-5p was able to inactivate the Wnt/β-catenin signaling pathway through directly targeting Wnt1.

RETRACTED

Several lncRNAs have been suggested to enhance or inhibit the Wnt/β-catenin signaling pathway during the development of cancer [42–44]. Pei et al demonstrated that down-regulation of lncRNA CASC2 remarkably promoted cell proliferation and metastasis of bladder cancer by activation of the Wnt/β-catenin signaling pathway [45]. However, the association between XIST and the Wnt/β-catenin signaling pathway in bladder cancer has not been studied. Our research revealed that knockdown of XIST significantly reduced expression levels of tumor-related genes (Wnt1, β-catenin and cyclin-D1) in the Wnt/β-catenin signaling pathway in bladder cancer cells. Furthermore, down-regulation of miR-139-5p could restore the repression of Wnt1, β-catenin and cyclin-D1 expressions induced by XIST knockdown. These results suggested that XIST regulated the Wnt/β-catenin signaling pathway in bladder cancer through miR-139-5p.

In summary, we demonstrated that lncRNA XIST was up-regulated in bladder cancer tissues and cell lines, and was correlated with worse survival of bladder cancer patients. In addition, XIST functioned as an oncogenic lncRNA that promoted cell growth and metastasis of bladder cancer through regulating miR-139-5p mediated Wnt/β-catenin signaling pathway. Therefore, these findings suggested that lncRNA XIST may serve as a potential therapeutic target for bladder cancer treatment.

## MATERIALS AND METHODS

### Clinical specimens

A total of 52 bladder cancer tissues and their matched adjacent non-tumor tissues were obtained from patients who underwent resection surgery at the Department of Urology, Gongli Hospital of the Second Military Medical University from 2008 to 2014. This study were approved by the Ethics Committee of Gongli Hospital of the Second Military Medical University and all the bladder cancer patients written informed consent to use the tissue samples for research purposes. All patients did not receive any treatment before the surgery. The clinicopathological characteristics of patients were recorded.

### Cell culture

Normal human urothelial cells (SV-HUC-1), bladder cancer cell lines (T24, 5637, EJ, UMUC3 and J82) and human embryonic kidney (HEK) 293T cells were obtained from the American Type Culture Collection (ATCC, Manassas, VA, USA). All cell lines were cultured in RPMI-1640 medium (Gibco, Carlsbad, CA, USA) supplemented with 10% fetal bovine serum (FBS), 100μg/ml streptomycin and 100U/ml penicillin at 37 °C in a humidified 5% CO2 incubator.

RETRACTED

### Cell transfection

Three short hairpin RNAs (shRNAs) targeting XIST (sh-XIST-1 sequences: 5'-GCCAACTGTCTGCTTAAGAAA-3', sh-XIST-2 sequences: 5'-GCTGCTAGTTTCCCAATGATA-3' and sh-XIST-3 sequences: 5'-GCGCGATAGCGCTAATAATTT-3'), negative control shRNA (sh-NC), miR-139-5p mimics, miR-139-5p inhibitor and negative control miRNA (miR-NC) were designed and constructed by GenePharma (Shanghai, China). Transfection was performed using Lipofectamine 2000 (Invitrogen, USA) according to the manufacturer’s instructions.

### RNA extraction and quantitative real-time PCR

The total RNA were extracted from clinical tissues or cell lines with Trizol reagent (Invitrogen, Carlsbad, USA) according to the manufacturer’s instructions. Total RNA were firstly reverse transcribed to cDNA using the PrimeScript RT Reagent Kit (Takara, Japan). Quantitative real-time PCR (qRT-PCR) was then performed with the SYBR Green PCR Kit (Takara, Japan) on the ABI 7500 Fast Real-Time PCR system (Applied Biosystems, CA, USA) following the instructions. Results were normalized to GAPDH and U6 respectively. The PCR primers were designed and synthesized by GenePharma (Shanghai, China). The primer sequences were as follows: XIST: 5'-ACGCTGCATGTGTCCTTAG-3' (forward) and 5'-GAGCCTCTTATAGCTGTTTG-3' (reverse); miR-139-5p: 5'-GCCTCTACAGTGCACGTGTCTC-3' (forward) and 5'-CGCTGTTCTCATCTGTCTCGC-3' (reverse); Wnt1: 5′-CCCTAACCGGTGCGCCCTGGTGCC-3′ (forward) and 5′-AGCGCCCAGAGCCCCATGGCCTGC-3′ (reverse). The relative expression levels of genes were calculated with the 2^-ΔΔCt^ method.

### CCK-8 assay

Cell proliferation was determined by Cell Counting Kit-8 assay (CCK-8, Beyotime, China). Briefly, T24 and 5637 cells were seeded into a 96-well plate. 48h after transfection, CCK-8 reagent was added into each well and further incubated for 1h. The absorbance at the wavelength of 450 nm was finally evaluated by a microplate reader.

### Colony formation assay

Transfected cells were plated in a six-well plate and incubated in DMEM medium supplemented with 10% FBS. 14 days later, the cells were fixed with 4% formaldehyde and then stained with 0.2% crystal violet (Sigma, USA). The number of colonies was counted and analyzed.

### Cell cycle assay

The transfected cells were harvested for cell cycle analysis at 48h after transfection. Cells were then fixed with 70% cold anhydrous ethanol at 4 °C for 2h before being stored at -20 °C. The fixed cells were washed and incubated with propidium iodide (PI, Sigma, USA) in the presence of RNase A at room temperature for 30min. The cell cycle distribution was immediately analyzed by flow cytometer equipped with Cell Quest software (FACSCalibur, BD Biosciences, USA).

RETRACTED

### Cell apoptosis assay

The transfected cells were harvested after transfection for 48h. Cell apoptosis was determined by the FITC-Annexin V apoptosis detection kit (BD Biosciences, USA) according to manufacturer’s instructions. After double staining by FITC-Annexin V and PI, the results were analyzed using flow cytometer (FACSCalibur, BD Biosciences, USA).

### Transwell migration and invasion assay

The migratory and invasive abilities of bladder cancer cells were evaluated by a transwell filter (pore size, 8μm; BD Biosciences). For cellinvasion assay, the membrane was coated with Matrigel (BD, NJ, USA) to form a matrix barrier. Transfected cells were suspended in serum-free medium and added to the upper chamber. Complete medium was added to the matched lower chamber as chemoattractant. After incubation for 24h, cells on the upper surface were removed with a cotton swab, and cells that had migrated to the bottom surface of the filter membrane were fixed with 4% formaldehyde, then stained with 0.1% crystal violet. The number of migration and invasion cells were photographed and counted in five randomly selected fields using a light microscope.

### Western blot analysis

Cells were lysed with the RIPA protein extraction reagent, and concentrations of protein were detected using a BCA Protein Assay Kit (Beyotime, Shanghai, China). Equal amounts of protein were separated by 10% SDS-PAGE, and then transferred to the PVDF membrane. The membranes were blocked with 5% non-fat milk for 1h, incubated with primary antibodies against Wnt1, β-catenin, cyclin-D1 and GAPDH (with dilution of 1:800, 1:500, 1:800, 1:1000, respectively) (Abcam, MA, USA) at 4°C overnight, and followed by incubation with HRP-conjugated secondary antibodies (Abcam, MA, USA) at room temperature for 2h. The results were finally analyzed by using the ECL detection system (Pierce Biotechnology, Rockford, USA) according to manufacturer’s instructions.

### Luciferase reporter assays

The wild-type and mutant XIST containing the binding site of miR-139-5p were inserted into the pmirGLO dual-luciferase vector to form the reporter vector XIST-wild-type (XIST-WT) and XIST-mutant (XIST-MUT). HEK293T cells were then co-transfected with XIST-WT or XIST-MUT, and miR-139-5p mimics by Lipofectamine 2000. 48h after transfection, the relative luciferase activities were measured with Dual-luciferase Reporter Assay System (Promega, USA) according to the manufacturer’s instructions. Similarly, the wild-type and mutant Wnt1 containing the binding site of miR-139-5p were incorporated into the pmirGLO dual-luciferase vector to form the reporter vector Wnt1-wild-type (Wnt1-WT) and Wnt1-mutant (Wnt1-MUT). The Wnt1-WT or Wnt1-MUT and miR-139-5p mimics were co-transfected into HEK293T cells. The relative luciferase activities were detected as described above.

RETRACTED

### RNA pull-down assay

The DNA fragment containing the miR-139-5p seed region binding site of XIST was PCR-amplified by using a T7-containing primer and then cloned into GV394 (GenePharma, Shanghai, China). Biotin-labeled RNAs were *in vitro* transcribed with the Biotin RNA Labeling Mix (Roche Diagnostics, USA) and T7 RNA polymerase (Takara Biomedical Technology, Japan). The products were treated with RNase-free DNase I and purified with the RNeasy Mini Kit (Qiagen, Valencia, CA, USA) according to manufacturer’s instructions. Whole-cell lysates was incubated with purified biotinylated XIST at room temperature for 1h, complexes were isolated with streptavidin agarose beads (Invitrogen, USA). The miR-139-5p present in the pull-down material was quantified by qRT-PCR.

### *In vivo* tumorigenesis assays

Four-week-old female athymic BALB/C nude mice were all purchased from Shanghai Experimental Animal Center of Chinese Academy of Sciences (Shanghai, China). The T24 cells transfected with XIST shRNA or negative control were subcutaneously injected into nude mice. Tumor volumes were examined weekly and calculated according to the following formula: tumor volume (mm^3^) = 0.5×length×width^2^. All nude mice were euthanized 6 weeks after injection and tumor weights were measured. The animal experiments were performed following the approval by the Animal Care and Experiment Committee of Gongli Hospital affiliated to the Second Military Medical University.

### Immunohistochemistry analysis

Tumor tissues from nude mice were fixed in 10% formalin and embedded with paraffin. Tissue sections were then deparaffinized by xylene and dehydrated in alcohol. Endogenous peroxidase activity was inhibited by 0.3% hydrogen peroxide for 30 min at room temperature. To block the sections, 5% bovine serum albumin in PBS was used for 1 h at room temperature. The sections were next incubated with rabbit polyclonal primary antibody against the cell proliferation marker Ki-67 (Abcam, USA) overnight at 4°C. Following washing with PBS, sections were incubated with secondary antibody for 1 h at room temperature. The products were assessed using a microscope (×200).

### Statistical analysis

All data were presented as the mean ± SD from three independent experiments. Differences between groups were analyzed by SPSS 20.0 software (SPSS, Chicago, USA) with the chi-square test, Student’s t-test or one-way ANOVA analysis. The relationship between the expressions of XIST, miR-139-5p and Wnt1 in clinical tissues was assessed by Pearson’s correlation analysis. Overall survival was evaluated by the Kaplan-Meier survival analysis with the log-rank test for comparison. P < 0.05 was considered statistically significant.
